# Two Uncommon Presentations of COVID-19-Associated Mucormycosis

**DOI:** 10.7759/cureus.21229

**Published:** 2022-01-14

**Authors:** Roger Rathna, Christopher D'Souza, Carol D'Silva, Jethin M Joseph, Athul K Varghese

**Affiliations:** 1 Critical Care Medicine, St. John's Medical College Hospital, Bangalore, IND; 2 General Medicine, St. John's Medical College Hospital, Bangalore, IND

**Keywords:** covid-19-associated mucormycosis, cutaneous mucormycosis, pulmonary mucormycosis, gastropleural fistula, fournier's gangrene

## Abstract

Mucormycosis is a rare opportunistic fungal infection commonly affecting immunocompromised individuals. There has been a surge in the number of these cases during the second wave of the Coronavirus Disease 2019 (COVID-19) in India. Mucormycosis has been reported to occur concurrently or a few weeks post-recovery from COVID-19. There have been multiple case reports/case series of rhino-orbital mucormycosis in India as a complication in COVID-19 pneumonia. We report two unique presentations of COVID-19-associated mucormycosis (CAM) in patients recently recovered from COVID-19. The first patient is an uncontrolled diabetic with Fournier’s gangrene at presentation, which on further evaluation, showed features of mucormycosis. The second one is a case of uncontrolled diabetes with a previous COVID-19 infection presenting with pulmonary mucormycosis and aspergillosis, complicated by a gastropleural fistula. While liposomal amphotericin B (L-ampB) was started for both patients, they significantly deteriorated during their course of hospital stay due to the severity of the disease.

## Introduction

Mucormycosis is most commonly caused by the genera in the order Mucorales. They are ubiquitous in nature, yet the rarity of acquiring the infection indicates the immune system's effectiveness. These infections were described as early as the 1800s, but have recently gained importance due to changing therapeutics with regard to immunosuppression, more so in the wake of the Coronavirus Disease 2019 (COVID-19) pandemic. The infection can present in many different ways in affected individuals, which is why their detailed description is essential.

## Case presentation

Case 1

A 47-year-old male, newly detected diabetic (glycosylated hemoglobin = 16.3%), was admitted with a background history of recovered mild COVID-19 infection one month ago, treated with steroids and anticoagulants. Three weeks post-recovery from COVID-19, he developed a fever of four-days duration and weakness of bilateral lower limbs. The weakness was sudden in onset, symmetrical, progressive, and associated with numbness and bowel and bladder incontinence. Simultaneously, he also noticed a skin discoloration on the dorsal surface of the penis, which slowly progressed to gangrenous changes and difficulty in micturition.

He first got admitted to a local hospital with these complaints, where he underwent penile debridement and a suprapubic cystostomy. He was also detected with diabetic ketoacidosis and hypokalemia at the time of admission and was treated for the same. An MRI spine was done, following which he was diagnosed with transverse myelitis. A pulse dose of pulse methylprednisolone (500 mg) was given over three days for the same. One week after staying in this hospital, the patient was referred to our center. He was on a postoperative day (POD) five at admission, following penile debridement with a suprapubic catheter (SPC) in situ. There were also complaints of decreased urine output since the last day prior to admission. On arrival at the ER, he was conscious, oriented, and hemodynamically stable. His neurological examination showed reduced sensations (pain, touch, and temperature) of his bilateral lower limbs and complete loss of sensations at the sole of both feet, reduced power in both lower limbs, with bowel and bladder incontinence. Deep tendon and plantar reflexes were mute. Other examination findings were unremarkable. Initial evaluation revealed that he was acidotic with capillary blood sugars upwards of 300 mg/dL.

He was admitted to a high dependency unit, where he received antibiotics and treatment for diabetic ketoacidosis. Despite adequate IV hydration, he went into oliguric acute kidney injury with increased serum creatinine to 2.53 mg/dL from a baseline of 0.8 mg/dL. Consults were sought from nephrology, urology, and plastic surgery departments. An MRI showed a disc bulge at the level of L3-L5 spinal roots, causing compression of the anterior thecal sac. After consultation with neurology, he received the remaining two doses of his five-day pulse steroid regimen with 1 gm methylprednisolone. He was shifted to the ICU for dialysis and hemodynamic monitoring dialysis. In the ICU, he underwent three sessions of hemodialysis. Penile gangrene with a clear line of demarcation in the junction of the upper 1/3rd and lower 2/3rd of the penile tissue was noted. The initial tissue swab from the penile site showed aseptate hyphae. The patient was initiated on liposomal amphotericin at a 3 mg/kg dose due to a strong suspicion of penile mucormycosis. A grade 3 bedsore over the sacral region was also noted. Due to persistent fever spikes and slough present at the penile wound, he underwent a total penectomy and partial scrotal closure. The tissue biopsy confirmed features of angioinvasive mucormycosis (Figure 1).

**Figure 1:** Grocott's methenamine silver stain of the penectomy specimen showing features (red arrows) of Mucormycosis.

Following the above surgeries, the Fournier's gangrene continued to extend to his perianal region, with blackish discoloration of the sacrum. Upon surgical consultation, he was taken up for another debridement for Fournier's gangrene and sacral bedsore, with a sigmoid colostomy three days later. Following the debridement, a contrast-enhanced computed tomography (CECT) abdomen was done. The imaging revealed Fournier's gangrene post-debridement with involvement of perineum, emphysematous cystitis, proctitis, and intramedullary air foci within the sacrum s/o osteomyelitis (Figure 2). 

**Figure 2:** A contrast-enhanced CT of abdomen showing intramedullary air foci within the sacrum (red arrow).

An interdepartmental meeting was held between general surgery, plastic surgery, and urology teams. It was opined that further debridements might be required due to the spread of the infection between the muscle planes. However, the surgical options were limited due to fulminant sepsis and poor general condition. The proposed surgical treatment was extensive, which included removing the rectum, gluteal muscles, and affected bony areas due to existing evidence of osteomyelitis. The family was unwilling to carry on further surgical treatment but wished for the medical management to continue. He was continued on liposomal amphotericin B and other broad-spectrum antibiotics. The patient's overall general condition continued to deteriorate with worsening septic shock, anemia, and thrombocytopenia. Due to the poor prognosis, the patient's family decided to discharge him against medical advice.

**Case 2**

The second case is of a 48-year-old male, diabetic (glycosylated hemoglobin = 10.6%), on oral hypoglycemic agents. He had a history of COVID-19 infection one month ago. He was treated with steroids, anticoagulants, and antibiotics at that time. Two weeks post COVID recovery, he developed chest pain and cough of one-week duration. A CT chest done in an outside hospital revealed a left-sided pyopneumothorax. An intercostal drain (ICD) was inserted for the same. He was referred to our hospital for a possible need for a thoracotomy. A repeat CT done in our hospital showed complete left lower lobe consolidation with segmental consolidation of the upper lobe, a probable superadded infection with ruptured cavitary transformation in the left upper lobe, left moderate hydropneumothorax, with ICD in situ and soft tissue emphysema. Also noted were left emphysematous pyelonephritis, splenomegaly with thyromegaly, and fatty liver. At admission, the patient had nonoliguric acute kidney injury (AKI). He underwent left double J (DJ) stenting for the emphysematous pyelonephritis, following which the AKI gradually resolved. A pleural fluid analysis done showed growth of Burkholderia and Enterococcus, for which relevant antibiotics were started. The patient had recurrent fever spikes. A repeat pleural fluid culture was done, which showed mucormycosis. Liposomal amphotericin at a dose of 5 mg/kg a day was started. On the fourth day of ICU stay, the ICD drain output showed ingested food particles approximately 15 minutes after patients' oral feed. A repeat CECT chest and abdomen revealed a gastropleural fistula and pleurocutaneous fistula (Figures 3-4).

**Figure 3:** A transverse section of a contrast-enhanced CT showing oral contrast extravasation (red arrow) into the left pleural space, indicating a fistulous opening from the GI tract into the pleural space.

**Figure 4:** A coronal section of contrast-enhanced CT showing oral contrast extravasation (red arrow) into the left pleural space, indicating a fistulous opening from the GI tract into the pleural space.

After consultation with the gastro surgery department, a feeding jejunostomy (FJ) and a closure of the fistula were planned. In view of increasing subcutaneous emphysema and chest wall cellulitis, a cardiothoracic surgery opinion was taken, and a new ICD was positioned and planned for debridement. The patient underwent thoracotomy and debridement with partial necrosectomy of the lung tissue, bullectomy, and bronchial stapling with FJ. The ICDs placed intraoperatively showed bile in the drain fluid persistently. The biopsy of the lung tissue showed mucormycosis with angioinvasion and invasive aspergillosis (Figure 5).

**Figure 5:** Lung biopsy showing broad aseptate hyphae (red arrows) confirmatory of mucormycosis.

In view of persistent bile leak from the ICD, he was posted for a laparotomy and closure of the gastropleural fistula. Preoperatively, an upper GI endoscopy was performed, which revealed a necrotic exudate in the lower esophagus and in the posterior wall of the proximal gastric body. A repeat CT done showed the same findings as before but with an increase in the pneumothorax, the left pararenal collection, and hepatosplenomegaly with suspected splenic infarct/evolving abscess. The patient was planned for a laparotomy to repair gastropleural fistula with partial gastrectomy, re-exploration for emphysematous pyelonephritis, and a possible pneumonectomy at a later date. The patient and his relatives were counseled about the prognosis, but as they were not willing for further surgical treatment, they sought discharge against medical advice.

## Discussion

Mucormycosis presents in different ways, especially in immunocompromised and diabetic individuals. Ninety percent of the cases present as rhino-orbital or rhino-orbito-cerebral mucormycosis, while the remaining 10% presents as pulmonary, cutaneous, or disseminated disease. Cutaneous presentations are sporadic [1]. CAM has been classified as early (within seven days of COVID-19 infection) and late (up to three months post-diagnosis of COVID-19 infection) [2]. We have described two unusual cases of CAM, one masquerading as Fournier's gangrene and the other as a case of pulmonary mucormycosis complicated by a gastropleural fistula. To the best of our knowledge, both of the above presentations have not been described up until now. Common to both was recent convalescence from COVID-19 infections, treatment with corticosteroids, and the presence of diabetes mellitus.

The possible etiologies for CAM that have been suggested are uncontrolled sugars with or without ketoacidosis, injudicious use of corticosteroids, hyperferritinemia, overexpression of glucose-regulated protein GRP78, and decreased phagocytic activity due to immunosuppression [1,2]. Long-term use of steroids is known to cause opportunistic infections like mucormycosis and aspergillosis. However, even a short course has been described to cause mucormycosis, especially in the diabetic population. In a new consensus definition for invasive fungal disease, a dose of ≥0.3 mg/kg corticosteroids for ≥3 weeks in the previous 60 days has been listed as a risk factor [3]. The use of glucocorticoids causes immune suppression and a hyperglycemic state. This accounts for a predilection to develop invasive fungal infections caused by Mucorales molds [4].

Severe COVID-19 infections have higher pro-inflammatory cytokine levels (IL-1, IL-2, IL-6, tumor necrosis alpha) and anti-inflammatory cytokine levels (IL-4, IL10), less CD4 interferon-gamma expression, and fewer CD4 and CD8 cells [5,6]. This also increases the risk for the development of invasive fungal infections like mucormycosis [6,7]. A complex interplay of agent, host, and environmental factors has been implicated in the surge of CAM during the second wave of COVID-19 in India. Pulmonary mucormycosis and disseminated mucormycosis have been associated with higher mortality. Overall, the reported mortality owing to CAM has been 36.5% [2]. The mainstay of treatment includes prompt surgical debridement and initiating antifungal therapy that includes amphotericin with or without posaconazole/isavuconazole. In both the cases discussed earlier, appropriate antifungal therapy was started, surgical interventions were done, and yet the disease continued to progress, indicating the seriousness of the issue.

## Conclusions

Pulmonary and cutaneous mucormycosis are less common presentations of this fatal disease. However, the mortality in these cases remains high despite appropriate medical and surgical therapy. Therefore, in the setting of the COVID-19, a high degree of suspicion, especially in patients who are diabetic or immunocompromised, is vital for early recognition and to avoid morbidity and mortality.
